The article "LncRNA PVT1 triggers Cyto-protective autophagy and promotes pancreatic ductal adenocarcinoma development via the miR-20a-5p/ULK1 Axis" was retracted in 2022. Reasons: manipulated images; duplicated images; lack of ethics approval or compliance; a breach of policy by an author.

# LncRNA PVT1 triggers Cyto-protective autophagy and promotes pancreatic ductal adenocarcinoma development via the miR-20a-5p/ULK1 Axis

**DOI:** 10.1186/s12943-018-0845-6

**Published:** 2018-07-12

**Authors:** Fengting Huang, Wenying Chen, Juanfei Peng, Yuanhua Li, Yanyan Zhuang, Zhe Zhu, Chunkui Shao, Wanling Yang, Herui Yao, Shineng Zhang

**Affiliations:** 1 Department of Gastroenterology and Guangdong Provincial Key Laboratory of Malignant Tumor Epigenetics and Gene Regulation, Sun Yat-sen Memorial Hospital, Sun Yat-sen University, No. 107 Yanjiang West Road, Guangzhou, 510120 China; 2 Department of Gastroenterology, Sun Yat-sen Memorial Hospital, Sun Yat-sen University, Guangzhou, 510120 China; 3 Department of Medicine, Division of Regenerative Medicine, University of California, San Diego, School of Medicine, La Jolla, CA 92093 USA; 4 Department of Pathology, The Third Affiliated Hospital, Sun Yat-sen University, Guangzhou, 510630 China; 5 Department of Paediatrics and Adolescent Medicine, Centre for Genomic Sciences, LKS Faculty of Medicine, The University of Hong Kong, Pokfulam, Hong Kong; 6 Department of Medical Oncology, Sun Yat-sen Memorial Hospital, Sun Yat-sen University, No. 107 Yanjiang West Road, Guangzhou, 510120 China

**Keywords:** Long non-coding RNA, PVT1, Autophagy, ULK1, miR-20a-5p, Pancreatic ductal adenocarcinoma

## Abstract

**Background:**

Defective autophagy is thought to contribute to the pathogenesis of many diseases, including cancer. Human plasmacytoma variant translocation 1 (PVT1) is an oncogenic long non-coding RNA that has been identified as a prognostic biomarker in pancreatic ductal adenocarcinoma, but how PVT1 operates in the regulation of autophagy in pancreatic ductal adenocarcinoma (PDA) is unclear.

**Methods:**

PVT1 expression level was detected by quantitative real-time polymerase chain reaction (qRT-PCR) and hybridization in situ (ISH). Western blot or qRT-PCR was performed to assess the ULK1 protein or mRNA level. Autophagy was explored via autophagic flux detection under a confocal microscope and autophagic vacuoles investigation under a transmission electron microscopy (TEM). The biological role of PVT1 in autophagy and PDA development was determined by gain-of-function and loss-of-function assays.

**Results:**

We found that PVT1 levels paralleled those of ULK1 protein in PDA cancer tissues. PVT1 promoted cyto-protective autophagy and cell growth by targeting ULK1 both in vitro and in vivo. Moreover, high PVT1 expression was associated with poor prognosis. Furthermore, we found that PVT1 acted as sponge to regulate miR-20a-5p and thus affected ULK1 expression and the development of pancreatic ductal adenocarcinoma.

The article "LncRNA PVT1 triggers Cyto-protective autophagy and promotes pancreatic ductal adenocarcinoma development via the miR-20a-5p/ULK1 Axis" was retracted in 2022. Reasons: manipulated images; duplicated images; lack of ethics approval or compliance; a breach of policy by an author.

**Conclusions:**

The present study demonstrates that the “PVT1/miR-20a-5p/ULK1/autophagy” pathway modulates the development of pancreatic ductal adenocarcinoma and may be a novel target for developing therapeutic strategies for pancreatic ductal adenocarcinoma.

**Electronic supplementary material:**

The online version of this article (10.1186/s12943-018-0845-6) contains supplementary material, which is available to authorized users.

## Background

Pancreatic ductal adenocarcinoma (PDA) is one of the most lethal diseases of all human malignancies worldwide and ranks sixth in cancer-related deaths in China [1, 2]. PDA has an overall 5-year survival rate of less than 6% because most patients develop locally advanced or distant metastatic disease at the time of diagnosis. Even the most advanced chemotherapeutics and targeted therapies offer only modest survival benefits [3]. Thus, the development of innovative targeted molecular therapies for this disease is urgently needed to improve the therapeutic outcome of PDA.

Recently, long non-coding RNAs (lncRNAs) have attracted widespread attention due to their potential roles in development and diseases, including cancer [4]. lncRNAs comprise a heterogeneous family of RNA molecules longer than 200 nucleotides with no or limited protein-coding potential. Aberrant lncRNA expression has been observed in various types of cancers [5]. An increasing number of lncRNAs have recently been reported to play an important role in the carcinogenesis and development of PDA [6–9]. Multiple lncRNAs are involved in a variety of biological processes, including cell proliferation, metastasis, autophagy and apoptosis. These data imply that lncRNAs may represent a new class of PDA biomarkers and therapeutic targets.

Human plasmacytoma variant translocation 1 (PVT1), a long intergenic non-coding RNA homologous to the mouse plasmacytoma variant translocation gene [10], has been found to map to chromosome 8q24, a region with frequent copy number amplification [11]. Amplification of PVT1 is one of the most frequent events in human digestive system tumors, including hepatocellular carcinoma [12], gastric cancer [13, 14], and colorectal cancer [15, 16]. The high expression of PVT1 in these tumors is indicative of poor prognosis. Consistent with these findings, PVT1 is dysregulated and associated with clinical stage and patient outcomes in PDA [17]. A previous genome-wide association study (GWAS) identified a PVT1 susceptibility locus at 8q24.21 (rs1561927) that is associated with risk of PDA [18]. In addition, in the human pancreatic cancer cell line AsPC-1, functional inactivation of the PVT1 gene can enhance gemcitabine sensitivity, whereas ectopic expression of PVT1 reverses this effect [19]. Collectively, various studies have clearly revealed that PVT1 plays an important role in carcinogenesis and chemoresistance. However, the functional roles and mechanisms of PVT1 in PDA remain poorly understood, and thus need to be further elucidated.

The article "LncRNA PVT1 triggers Cyto-protective autophagy and promotes pancreatic ductal adenocarcinoma development via the miR-20a-5p/ULK1 Axis" was retracted in 2022. Reasons: manipulated images; duplicated images; lack of ethics approval or compliance; a breach of policy by an author.

MicroRNAs (miRNAs) are endogenous RNAs of approximately 23 nucleotides in length that play important roles in almost all biological activities [20]. miRNAs have also emerged as major players in the cancer paradigm, with potential effects in both oncogenic and tumor-suppressive pathways [21]. miRNAs are well known to regulate gene expression at the posttranscriptional level. Moreover, new regulatory circuitry has been revealed in which RNAs can interact with each other by competing for shared miRNAs. Such competing endogenous RNAs (ceRNAs) affect the distribution of miRNAs and subsequent target gene expression [22]. A number of studies have shown that some lncRNAs can act as ceRNAs through their miRNA-binding sites [23–25], raising questions as to whether PVT1 also involves in similar crosstalk with miRNAs.

In the present study, we found that PVT1 levels paralleled with ULK1 (Unc-51 like kinase 1) protein expression, a key molecule involved in triggering autophagy initiation, in PDA. PVT1 promoted cyto-protective autophagy and cell growth both in vitro and in vivo. Furthermore, we found that PVT1 acts as sponge to regulate miR-20a-5p and thus affects ULK1 expression. Taken together, our results demonstrate that the “PVT1/miR-20a-5p/ULK1/autophagy” pathway modulates the development of PDA, indicating that this pathway is a novel target for developing therapeutic strategies to treat PDA.

## Methods

### Gene expression omnibus (GEO) and the Cancer genome atlas (TCGA) analysis

PDA patient gene profiling data were downloaded from the National Center for Biotechnology Information GEO database (GSE15471 and GSE16515) (https://www.ncbi.nlm.nih.gov/) and The Cancer Genome Atlas (TCGA) Data Portal (https://tcga-data.nci.nih.gov/tcga/). We utilized UCSC hg19 as the *Homo sapiens* reference genome and gene model for read mapping and quantification.

### Cell lines

PDA cell lines (HPAF-II, PANC-1, SW1990, BxPC-3, MIA PaCa-2, Capan-2 and AsPC-1) were purchased from American Type Culture Collection (ATCC, Rockville, MD, USA) and cultured in RPMI1640 medium (Invitrogen, Carlsbad, CA, USA) supplemented with 10% fetal bovine serum (FBS). The immortalized pancreatic ductal epithelial cell line H6C7, a gift from Prof. Ming-Sound Tsao of the Ontario Cancer Institute (Ontario, Canada), was incubated in keratinocyte serum-free medium (Invitrogen) containing 1% penicillin/streptomycin, 0.2 ng/ml recombinant endothelial growth factor and 20 ng/ml bovine pituitary extract. The HEK 293 T cell line was obtained from ATCC (Rockville, MD, USA) and cultured in Dulbecco’s modified Eagle’s medium (Invitrogen) supplemented with 10% FBS. For autophagy detection, cells were incubated with either an autophagy inhibitor (3-methyladenine, 3-MA, 5 mmol/L, Sigma-Aldrich) or an autophagy inducer (rapamycin, 2 μmol/L, Sigma-Aldrich). All cells were maintained at 37 °C in a humidified 5% CO_2_ atmosphere.

The article "LncRNA PVT1 triggers Cyto-protective autophagy and promotes pancreatic ductal adenocarcinoma development via the miR-20a-5p/ULK1 Axis" was retracted in 2022. Reasons: manipulated images; duplicated images; lack of ethics approval or compliance; a breach of policy by an author.

### Clinical specimens

PDA specimens and adjacent non-tumor tissues were obtained from patients undergoing surgery at Sun Yat-sen Memorial Hospital. All specimens were derived from patients who had not undergone chemotherapy or radiotherapy before surgery. Patient clinicopathological characteristics are summarized in Additional file 1: Table S1. The protocols used in the present study were approved by the Ethics Committee of Sun Yat-sen Memorial Hospital.

### Quantitative real-time polymerase chain reaction (qRT-PCR)

Total RNA was isolated from tissues or cultured cells using Trizol reagent (Invitrogen) according to the manufacturer’s protocol. One microgram of total RNA was reverse transcribed in a final volume of 20 μl using PrimeScript RT Master Mix (Takara, Dalian, China). qRT-PCR was performed as described previously [26]. Primer sequences are listed in Additional file 1: Table S2.

### Subcellular fractionation

To determine the cellular localization of PVT1, cytoplasmic and nuclear RNA were isolated using PARIS Kit (Life Technologies, MA, USA) according to the manufacturer’s instructions. GAPDH and U6 were used as markers of the cytoplasm and nucleus, respectively, in qRT-PCR.

### In situ hybridization

To explore the expression pattern of PVT1 in PDA, in situ hybridization was conducted with double Digoxigenin-labeled probes (Exiqon, vedbaek, Denmark) according to the manufacturer’s instruction. Briefly, the PDA tissues were sectioned at 4 μm thick and deparaffinized, then treated with proteinase-K (20 μg/ml) for 10 min at 37 °C. Slides were prehybridizated with the 1 × ISH buffer (Exiqon) and then hybridizated with digoxigenin-labeled probes at 45 °C for 1 h. Afterwards, the slides were incubated with anti-digoxigenin antibody (Roche Diagnostics, IN) at 4 °C overnight, and then stained with nitro blue tetrazolium/5-bromo-4-chloro-3-indolyl phosphate. The sequences of the probes are as follows: PVT1 probe: 5’-AACAGGGCAGGATCTATGGCAT-3′ and scramble probe: 5’-GTGTAACACGTCTATACGCCCA-3′.

### Plasmid and lentivirus constructs

Two small hairpin RNA (shRNA) sequences (GenePharma, Shanghai, China) were used to construct a PVT1-shRNA lentivirus (LV-shPVT1–1 and LV-shPVT1–2) (GenePharma) as reported previously [27]. The efficacy was detected by qRT-PCR and a scrambled shRNA was used as a negative control and named LV-shNC. To generate a PVT1 expression vector, full-length human PVT1 (NR_003367) was synthesized and subcloned into the pGLV3/H1/GFP/Puro plasmid (GenePharma) for lentivirus production and named LV-PVT1. An empty vector containing the green fluorescent protein was used as a negative control for LV-PVT1 and named LV-NC. All shRNA sequences are listed in Additional file 1: Table S3.

The article "LncRNA PVT1 triggers Cyto-protective autophagy and promotes pancreatic ductal adenocarcinoma development via the miR-20a-5p/ULK1 Axis" was retracted in 2022. Reasons: manipulated images; duplicated images; lack of ethics approval or compliance; a breach of policy by an author.

### Cell growth assay

For the MTS assay (CellTiter 96 AQueous One Solution Cell Proliferation Assay), 1.5 × 10^3^ cells per well were cultured in 96-well plates and detected at the indicated time-point using a cell counting kit (Promega, Madison, WI, USA). The 5-ethynyl-2′-deoxyuridine (EdU) immunofluorescence staining was performed using the EdU kit (RiboBio, Guangzhou, China) according to the manufacturer’s protocol. For the colony-formation assay, cells were harvested, dissociated into single-cell suspensions and seeded in 6-well plates (2 × 10^3^ cells per well). The medium was replaced every 3 days. After 14 days, colonies (> 50 cells/colony) were stained with Giemsa, counted, and photographed. Each experiment was performed in triplicate.

### Flow cytometric analysis

Cell cycle and apoptosis analysis was detected by flow cytometric assay. Flow cytometric analysis was conducted as previously described [27].

### Western blotting

Cell lysates were prepared as described previously [27]. Equal amounts of proteins obtained from different kinds of cell lysates were separated by 10% or 15% SDS-PAGE, transferred to PVDF membranes, and subjected to western blotting using an ECL chemiluminescence reagent (GE Healthcare). Antibodies for ULK1 (ab128859), LC3b (ab192890) and GAPDH (ab9485) were purchased from Abcam (Cambridge, MA, USA).

### Immunohistochemistry

Immunohistochemistry for the target molecules was performed on paraffin sections using primary antibodies against Ki67 (#9449, Cell Signaling Technology, Danvers, MA, USA) and ULK1 (ab128859, Abcam, Cambridge, MA, USA), as well as horseradish peroxidase-conjugated IgG, and proteins were visualized in situ with 3, 3-diaminobenzidine kit (BioGenex, Fremont, CA, USA).

### Autophagy detection

2 × 10^4^ cells per well were seeded into 6-well plate and cultured in complete medium. Autophagy detection using mRFP-GFP-LC3 adenoviral vectors, which were purchased from HanBio Technology Co. Ltd. (HanBio, shanghai, China). Adenoviral infection was conducted according to the manufacturer’s instructions. Briefly, cells were plated and infected with the adenoviruses at a MOI of 300 for 5.5 h at 37 °C. After incubation with a fresh complete medium for 20 h, cells were transfected with LV-PVT1 or LV-NC. Autophagy was investigated under a confocal microscope Zeiss LSM 710 (Zeiss, Oberkochen, Germany). Images were acquired on the confocal microscope using a 63 x lens. The acquisition setting was set between samples and experiments to: XY resolution = 1024 × 1024 pixels, pinhole adjusted to 1.1 μm of Z thickness, increments between stack images were 1 μm, laser power and gain were set for each antibody. Autophagic flux was determined by calculating the number of GFP and mRFP dot (dots/cell were counted).

The article "LncRNA PVT1 triggers Cyto-protective autophagy and promotes pancreatic ductal adenocarcinoma development via the miR-20a-5p/ULK1 Axis" was retracted in 2022. Reasons: manipulated images; duplicated images; lack of ethics approval or compliance; a breach of policy by an author.

### Transmission electron microscopy (TEM)

TEM was performed according to the instruction carried out previously [28]. Briefly, cells were washed in phosphate buffered saline (PBS) and fixed in 2.5% glutaraldehyde and further fixed with 1% osmium tetroxide buffer, dehydrated using a graded ethanol series and embedded in 812 resin. Ultrathin sections were stained with aqueous uranyl acetate and lead citrate. The number of autophagic vacuoles was determined for a minimum of 100 cells, and the autophagic vacuoles were photographed on a JEM-100CX-II TEM (Joel, Tokyo, Japan) at 80 kV.

### Luciferase reporter assay

The human PVT1 3’UTR luciferase reporter construct (PVT1-wt) was generated by cloning the PVT1 mRNA 3’UTR sequence downstream of the psiCHECK luciferase reporter vector (Promega). The miR-20a-5p target site-mutation PVT1 3’UTR luciferase reporter (PVT1-mut) construct was generated using the QuikChange II XL Site-Directed Mutagenesis Kit (Stratagene, La Jolla, CA, USA). Wild-type ULK1 (ULK1-wt) and the mutant derivative devoid of the miR-20a-5p binding site (ULK1-mut) were cloned downstream of the luciferase gene coding sequence. The nucleotide sequences of all constructs were confirmed by DNA sequencing. Luciferase reporter plasmids plus miR-20a-5p mimics or miR-NC were co-transfected into HEK 293 T and HPAF-II cells using Lipofectamine 2000 (Invitrogen). Relative luciferase activity was measured as described previously [27]. All experiments were performed in triplicate. The primers used are listed in Additional file 1: Table S2.

### Animal models

Animal studies were approved by the Institutional Animal Care and Use Committee of Sun Yat-sen University, Guangzhou, China. Male athymic BALB/c nude mice (4–5 weeks old) were used for animal studies. The mice were kept in pathogen-free conditions. A total of 1 × 10^7^ HPAF-II cells stably transfected with LV-shPVT1–1, LV-shPVT1–2 or LV-shNC were subcutaneously injected into nude mice to generate xenografts. Xenograft growth was monitored using the in vivo fluorescence imaging system (IVIS) (Caliper Life Sciences, Hopkinton, MA), and the size and weight of the xenografts were measured periodically. For the IVIS, tumors that developed in xenograft-transplanted mice were viewed and the luciferase signals were captured 10 min after vein injection with 100 μl of 50 nM nano-luciferin (Promega). The tumor volume was calculated according to the following equation: volume = length × width^2^ × 0.5.

The article "LncRNA PVT1 triggers Cyto-protective autophagy and promotes pancreatic ductal adenocarcinoma development via the miR-20a-5p/ULK1 Axis" was retracted in 2022. Reasons: manipulated images; duplicated images; lack of ethics approval or compliance; a breach of policy by an author.

### Terminal dexynucleotidyl transferase(TdT)-mediated dUTP nick end labeling (TUNEL) assay

To investigate the apoptosis in xenograft PDA model, TUNEL (Roche) assay was carried out according to the manufacturer’s instruction, as described earlier [27].

### RNA pull-down assay

RNA pull-down assays were performed as described previously [29]. Briefly, PVT1-sense and PVT1-antisense were in vitro transcribed from vector pGEM-T-PVT1, biotin-labeled using the Biotin RNA Labeling Mix and T7 RNA polymerase (Thermo Fisher Scientific), treated with RNase-free DNase I (Thermo Fisher Scientific), and purified with an RNeasy Mini Kit (Qiagen, Valencia, CA, USA). One milligram of whole-cell lysate from HPAF-II cells was incubated with probe-coated beads, and after washing with wash/binding buffer, the RNA complexes bound to the beads were eluted and extracted for qRT-PCR analysis.

### RNA-binding protein immunoprecipitation (RIP) assay

RIP assays were performed using the Magna RIP Kit (Millipore, Bedford, MA, USA) according to the manufacturer’s instructions. Briefly, cells were lysed in complete RIP lysis buffer, and cell extracts were incubated with RIP buffer containing magnetic beads conjugated with human anti-AGO2 antibody or negative control normal mouse IgG. The retrieved RNA was then detected by qRT-PCR. U6 was used as a non-specific control.

### Statistical analysis

Statistical analyses were performed using SPSS 17.0 software (SPSS, Chicago, IL, USA). All numerical data were presented as the means ± standard deviation for multiple samples. The chi-square test (*χ*^2^-test) for non-parametric variables and Student’s *t* test or one-way analysis of variance (ANOVA) for parametric variables were used (two tailed). Correlations between PVT1 and ULK1 or miR-20a-5p were analyzed by Pearson rank correlation. Survival was calculated using the Kaplan-Meier method and analyzed by the log-rank test. *P* < 0.05 was considered significant.

## Results

### ULK1 protein levels parallel PVT1 expression in a subset of human PDA tissues

Previous studies have demonstrated that ULK1 is a key molecule involved in triggering autophagy initiation [30] and is dysregulated in many cancers, including PDA [31]. To validate this phenomenon, we investigated ULK1 expression in 20 PDA tissues and their corresponding adjacent non-tumor tissues. As shown in Fig. 1a-b, ULK1 protein levels were elevated in 13 out of 20 PDA tissues compared with the corresponding non-tumor tissues. However, ULK1 mRNA levels did not differ significantly between PDA and adjacent non-tumor tissues (Fig. 1c), which was further confirmed by analyzing ULK1 mRNA expression in a large cohort of PDA patients using the TCGA database (Additional file 1: Figure S1a). Meanwhile, we found that PVT1 was dramatically up-regulated in 20 PDA tissues compared with the corresponding non-tumor tissues (Fig. 1d-e). Intriguingly, correlation analyses showed that ULK1 protein levels paralleled PVT1 levels in PDA tissues (Fig. 1f). In addition, compared with the immortalized pancreatic ductal epithelial cell line H6C7, PVT1 levels were significantly increased in a panel of cell lines, with the exception of Capan-2 and MIA PaCa-2 (Fig. 1g). And positive correlation between PVT1 and ULK1 protein was also observed in PDA cell lines (Fig. 1h, Additional file 1: Figure S1b). These results suggest that PVT1 expression might be positively associated with ULK1 protein level in PDA.

The article "LncRNA PVT1 triggers Cyto-protective autophagy and promotes pancreatic ductal adenocarcinoma development via the miR-20a-5p/ULK1 Axis" was retracted in 2022. Reasons: manipulated images; duplicated images; lack of ethics approval or compliance; a breach of policy by an author.

**Fig. 1:** ULK1 protein level parallels to that of PVT1 in a subset of human PDA tissues. **a** Western blot analysis of the expression of ULK1 protein in PDA tissues (*n* = 20) and the corresponding adjacent non-tumor pancreatic specimens (n = 20). GAPDH acted as an endogenous control. T, tumor tissues; N, non-tumor pancreatic tissues; **b** The quantitation of the western blot results in (a). ULK1 protein expression was up-regulated in 13 PDA tissues compared with the corresponding adjacent non-tumor pancreatic specimens in 20 PDA tissues. The high value of ULK1 protein was defined as fold change > 1 (*n* = 13); **c** The level of ULK1 mRNA in 20 PDA tissues was of no statistical significance compared to that of the corresponding adjacent non-tumor pancreatic specimens by qRT-PCR. Data are presented as the mean ± S.D. (n = 20); **d** PVT1 expression in PDA tissues from the 20 PDA cases based on qRT-PCR analysis. The high value of PVT1 was defined as fold change > 2 (*n* = 15), the rest including down-regulation or no evident difference in expression in PDA tissues compared with PDA expression in the corresponding adjacent non-tumor tissue, was defined as low values (*n* = 5); **e** PVT1 expression in PDA tissues based on ISH analysis and the percent of PVT1-positive samples in different groups; **f** The expression level of PVT1 mRNA was positively correlated with that of ULK1 protein in 20 PDA tissues. The statistical analysis was performed using Pearson’s correlation coefficient (*R* = 0.8659, *P* < 0.0001); **g** The level of PVT1 mRNA in PDA cell lines by qRT-PCR. GAPDH acted as an endogenous control; **h** The expression level of PVT1 mRNA was positively correlated with that of ULK1 protein in PDA cell lines (*R* = 0.8546, *P* = 0.0069). Data are presented as the mean ± S.D. from three independent experiments. ^*^P < 0.05, ^**^P < 0.01 by Student’s t-test

The article "LncRNA PVT1 triggers Cyto-protective autophagy and promotes pancreatic ductal adenocarcinoma development via the miR-20a-5p/ULK1 Axis" was retracted in 2022. Reasons: manipulated images; duplicated images; lack of ethics approval or compliance; a breach of policy by an author.

### PVT1 induces autophagy by up-regulating ULK1 protein in vitro

To explore the biological role of PVT1 in PDA autophagy, we first performed ectopic expression of PVT1 in Capan-2 and MIA PaCa-2 cells by transfected with full-length of PVT1 cDNA, and knocked down PVT1 expression in SW1990 and HPAF-II cells using two small hairpin RNAs (shRNAs). qRT-PCR showed that PVT1 was effective up-regulated (Fig. 2a) or knockdown (Fig. 2b). TEM analysis showed that enhanced expression of PVT1 increased autophagic vacuoles in Capan-2 and MIA PaCa-2 cells (Fig. 2c). In addition, diminished autophagic vacuoles were observed with down-regulation of PVT1 expression in SW1990 and HPAF-II cells (Fig. 2d). Meanwhile, because microtubule-associated protein 1 light chain 3 (MAP1LC3/LC3) is a specific marker of autophagy initiation, the accumulation of GFP-LC3 puncta provides an effective way to detect autophagosomes. Consistent with the TEM results, PVT1 overexpression induced increased GFP-LC3 numbers of punctate structures (Fig. 3a, c). Whereas, attenuation of PVT1 expression decreased the numbers of GFP-LC3 punctate (Fig. 3b, d). These data imply that PVT1 can induce autophagy in PDA cells in vitro.

**Fig. 2:** Regulation of PVT1 made contributions to autophagy in PDA cells. **a** PVT1 level was overexpressed by specific lentivirus transfection in Capan-2 and MIA PaCa-2 cells; **b** PVT1 level was markedly suppressed by specific sh-RNAs in SW1990 and HPAF-II cells; **c** The ultrastructure of cells with or without up-regulation of PVT1 in Capan-2 and MIA PaCa-2 cells was observed by transmission electron microscopy. Autophagic vacuoles were increased after overexpression of PVT1 in Capan-2 and MIA PaCa-2 cells. Scale bar, 2 μm; **d** The ultrastructure of cells with or without down-regulation of PVT1 in SW1990 and HPAF-II cells. Autophagic vacuoles were decreased after attenuation of PVT1 expression in SW1990 and HPAF-II cells. Scale bar, 1 μm. Data are presented as the mean ± S.D. (*n* = 3). ^*^P < 0.05, ^**^P < 0.01 and ^***^P < 0.001 by Student’s t-test

**Fig. 3:** Detection of GFP-LC3 puncta with or without regulation of PVT1. **a**, **b** Representative images of GFP-LC3 puncta in PVT1-overexpressed cells (Capan-2 and MIA PaCa-2) (**a**) and PVT1-downregulated cells (SW1990 and HPAF-II) (**b**); **c**, **d** Quantitation of GFP-LC3 puncta in PVT1-overexpressed cells (Capan-2 and MIA PaCa-2) (**c**) and PVT1-downregulated cells (SW1990 and HPAF-II) (**d**). Enhanced expression remarkably increased the number of GFP-LC3 puncta. Meanwhile, down-regulation of PVT1 decreased the number of GFP-LC3 puncta. Data are presented as the mean ± S.D. (*n* = 3). ^*^P < 0.05 and ^**^P < 0.01 by Student’s t-test

Furthermore, growth curve indicated that overexpression of PVT1 promoted PDA cell proliferation. Interestingly, inhibition of proliferation was observed with treatment of autophagy inhibitor (3-methyladenine, 3-MA). Meanwhile, repression of PVT1 prohibited PDA cell growth. Markedly, restoration of proliferation occurred with treatment of autophagy inducer (rapamycin, rapa) (Fig. 4a). In accordance with growth curve, colony formation assays showed that up-regulation of PVT1 triggered PDA cell growth, with attenuation of growth occurred when 3-MA was used, meanwhile, down-regulation of PVT1 suppressed PDA cell proliferation, with restoration of growth observed when rapamycin was used (Fig. 4b). Moreover, EdU positive cells, which represented mitotic S phrase cells, were increased with overexpression of PVT1 in Capan-2 cells. Intriguingly, the number of EdU positive cells was decreased after treatment of 3-MA. On the other hand, suppression of PVT1 expression declined the number of EdU positive cells, with rescue after incubation of rapamycin (Fig. 4c). The result of cell cycle analyzed by flow cytometry was in accordance with that of EdU assay (Fig. 4d). As expected, apoptosis was decreased after augmentation of PVT1 expression. However, increased apoptosis was observed when autophagy inhibited (Fig. 4e). Taken together, these data suggest that PVT1 induces cyto-protective autophagy in PDA.

The article "LncRNA PVT1 triggers Cyto-protective autophagy and promotes pancreatic ductal adenocarcinoma development via the miR-20a-5p/ULK1 Axis" was retracted in 2022. Reasons: manipulated images; duplicated images; lack of ethics approval or compliance; a breach of policy by an author.

**Fig. 4:** PVT1 played a vital role in cyto-protective autophagy and PDA cells growth in vitro. **a** MTS assay indicated that up-regulation of PVT1 enhanced cells growth in Capan-2 cells. Whereas, impairment of growth was observed after incubation with autophagy inhibitor (3-MA) (upper). Meanwhile, down-regulation of PVT1 suppressed cells growth in HPAF-II cells. However, restoration of growth occurred after treatment with autophagy inducer (rapamycin) (lower); **b** Colony formation assay implied that increased PVT1 expression promoted cells proliferation in Capan-2 cells. However, 3-MA diminished cells proliferation in PVT1-overexpresssed cells. On the other hand, decreased PVT1 expression inhibited cells proliferation in HPAF-II cells. But rescue of cells growth was observed after treatment with rapamycin; **c** Cell proliferation was investigated by EdU incorporation assays; **d** Cell cycle analysis indicated that the percentage of mitotic S phase cells was increased after overexpression of PVT1 in Capan-2 cells. Decreased percentage occurred after incubation with 3-MA. Decreased expression of PVT1 diminished S phase cells in HPAF-II cells. Rescue of S phase happened after induction of autophagy by rapamycin; **e** Apoptosis prohibited after up-regulation of PVT1 in Capan-2 cells. Inhibition of autophagy promoted apoptosis. Meanwhile, down-regulation of PVT1 contributed to apoptosis in HPAF-II cells. Autophagy induction by rapamycin diminished the effect of down-regulation of PVT1 to apoptosis. The data were represented as the means ± S.D. of three independent experiments in vitro*.* ^*^P < 0.05 by Student’s t-test

It has been reported that up-regulation of ULK1 triggers autophagy in PDA cells. We then explored whether PVT1 induced autophagy by regulating ULK1. As shown in Fig. 5a, increased expression of PVT1 markedly induced autophagy with enhanced expression of LC3b II. Meanwhile, diminished expression of PVT1 inhibited autophagy with suppressive expression of LC3b II (Fig. 5b). Interestingly, ULK1 depletion significantly attenuated the effect of PVT1 in autophagy (Fig. 5c), whereas, enhanced expression of ULK1 remarkably restored the defect of PVT1 in autophagy (Fig. 5d), indicating that PVT1 induces autophagy by up-regulating ULK1 protein expression.

**Fig. 5:** PVT1 made an effort on autophagy via regulation of ULK1. **a** Western blot analysis of LC3b in Capan-2 and MIA PaCa-2 cells with or without up-regulation of PVT1. It was observed that the level of LC3b II was enhanced after increase of PVT1 expression; **b** LC3b II expression was decreased after down-regulation of PVT1; **c** Western blot analysis of LC3b in PVT1 stable-expressed Capan-2 and MIA PaCa-2 cells with or without depletion of ULK1. Suppression of LC3b II expression was detected after depletion of ULK1; **d** LC3b II expression was rescued after restoration of ULK1 in PVT1-knowndown SW1990 and HPAF-II cells

### Effects of PVT1 levels on PDA tumor growth in vivo

To probe the effect of PVT1 on cancer cell dynamics in vivo, we established the xenograft tumor models in nude mice using HPAF-II cell line with or without stable knockdown of PVT1. Stably-transfected cells using a lentivirus vector to mediate PVT1 suppression in HPAF-II cells were designated as HPAF-II sh-PVT1–1, HPAF-II sh-PVT1–2, and its counterpart HPAF-II sh-NC. The cells were subcutaneously injected into the right armpits of nude BALB/c mice. Photomicrographs of the tumors showed that HPAF-II sh-PVT1 cells had lower growth potential than HPAF-II sh-NC cells (Fig. 6a-c). Down-regulating PVT1 significantly suppressed overall tumor growth (Fig. 6d-e). Furthermore, ULK1 or Ki67 staining was decreased in xenografts of HPAF-II sh-PVT1 cells compared with HPAF-II sh-NC cells. While increased number of TUNEL positive cells was observed after suppression of PVT1 (Fig. 6f-i). These results indicated that suppression of PVT1 attenuated the growth of PDA through its interaction with ULK1, consistent with the in vitro results.

The article "LncRNA PVT1 triggers Cyto-protective autophagy and promotes pancreatic ductal adenocarcinoma development via the miR-20a-5p/ULK1 Axis" was retracted in 2022. Reasons: manipulated images; duplicated images; lack of ethics approval or compliance; a breach of policy by an author.

**Fig. 6:** Knockdown of PVT1 prohibited PDA growth in vivo. **a** Down-regulation of PVT1 in HPAF-II cells inhibited tumor growth after 4 weeks in vivo (*n* = 5 per group). Upper: negative control group. Lower: knockdown groups formed in nude mice subcutaneously injected with PVT1-silencing HPAF-II cells; **b**, **c** Growth curves (**b**) and tumor weight (**c**) of xenograft tumors after subcutaneous injection with PVT1-silencing HPAF-II cells. The tumor volumes were investigated every week after injection with PVT1-silencing HPAF-II cells (*n* = 5). Diminished expression of PVT1 markedly attenuated the tumor growth in PDA; **d**, **e** Representative images (**d**) and photon influx (**e**) of xenograft tumors after subcutaneous injection with PVT1-silencing HPAF-II cells by IVIS (*n* = 5 per group). **f** Representative images of HE staining, TUNEL, immunohistochemical staining of Ki67 and ULK1; **g-i** The quantitation of Ki67 (**g**), TUNEL (**h**) and ULK1 (**i**) was calculated. Immunohistochemical staining of Ki67 and ULK1 showed that decreased expression of PVT1 led to suppression of Ki67 proliferation index and ULK1 expression, while TUNEL positive cells were increased. The data were represented as the mean ± S.D. (*n* = 5). ^*^P < 0.05, ^**^P < 0.01 and ^***^P < 0.001 by Student’s t-test

### PVT1 regulates ULK1 expression in a posttranscriptional manner

To identify the underlying mechanism responsible for PVT1 to regulate ULK1 expression, we ectopically expressed PVT1 in Capan-2 and MIA PaCa-2 cells. Interestingly, overexpression of PVT1 failed to up-regulate ULK1 mRNA (Additional file 1: Figure S2a) but markedly elevated ULK1 protein in Capan-2 and MIA PaCa-2 cells (Additional file 1: Figure S2b). To silence PVT1, two shRNAs (sh-PVT1–1 and sh-PVT1–2) were used. Silence of PVT1 had little effect on ULK1 mRNA (Additional file 1: Figure S2c) but significantly down-regulated ULK1 protein in HPAF-II and SW1990 cells (Additional file 1: Figure S2d). The above results indicated that PVT1 regulates ULK1 expression at the posttranscriptional level.

### PVT1 modulates ULK1 expression by sponging miR-20a-5p

We have demonstrated that PVT1 regulates ULK1 expression at the posttranscriptional level. It is well-known that miRNAs act as negative regulators of gene expression at the posttranscriptional level [22]. However, lncRNAs can protect mRNAs by functioning as competing endogenous RNAs (ceRNAs) through sponging their targeted microRNAs. Thus, to demonstrate whether PVT1 plays as a ceRNA, we first applied bioinformatics analysis to explore potential miRNAs targeting the ULK1 3’UTR (miRanda, PicTar and Targetscan, Additional file 1: Table S4) and targeting the PVT1 3’UTR (DIANA and StarBase v2.0, Additional file 1: Table S5). Based on these results, three miRNAs were identified (Fig. 7a). Then, we performed RNA pull-down to identify which miRNAs were involved in the interaction of PVT1. As shown in Fig. 7b, miR-20a-5p, miR-302a-3p and miR-17-5p were identified. Furthermore, we observed the ULK1 expression with overexpression or attenuation of these miRNAs expression in HPAF-II cells. Interestingly, among these miRNAs, miR-20a-5p markedly altered the expression of endogenous ULK1 (Fig. 7c). Moreover, RIP assays confirmed the specific interaction between PVT1 and miR-20a-5p in HPAF-II cells (Fig. 7d). We also detected the subcellular location of PVT1 and miR-20a-5p. PVT1 was expressed in both the cytoplasm and nucleus, while miR-20a-5p was mainly expressed in the cytoplasm (Additional file 1: Figure S3).

The article "LncRNA PVT1 triggers Cyto-protective autophagy and promotes pancreatic ductal adenocarcinoma development via the miR-20a-5p/ULK1 Axis" was retracted in 2022. Reasons: manipulated images; duplicated images; lack of ethics approval or compliance; a breach of policy by an author.

**Fig. 7:** PVT1 modulates ULK1 expression by sponging miR-20a-5p. **a** The venn diagram of common microRNAs targeting PVT1 3’UTR and ULK1 3’UTR. Three microRNAs were identified, including miR-20a-5p, miR-302a-3p and miR-17-5p; **b** PVT1 biotin pull down assay was performed. The level of target microRNAs in the pull down of biotin-labelled PVT1 or negative control was investigated and quantified by qRT-PCR in HPAF-II cells; **c** Western blot analysis of ULK1 expression in HPAF-II cells with or without overexpression (upper) or suppression (lower) of target microRNAs (miR-20a-5p, miR-302a-3p, miR-17-5p). Interestingly, overexpression of miR-20a-5p suppressed ULK1 protein expression most. While inhibition of miR-20a-5p promoted ULK1 protein expression effectively; **d** RIP assay and qRT-PCR were conducted to detect the enrichment of PVT1 and miR-20a-5p by using AGO2 antibody in HPAF-II cells. Non-immune IgG acted as an internal control. U6 was used as a non-specific control. Enhanced enrichment of PVT1 and miR-20a-5p with AGO2 antibody was observed compared with IgG; **e** Bioinformatics prediction of miR-20a-5p binding sites in PVT1 3’UTR sequence using Starbase or ULK1 3’UTR sequence using TargetScan was presented; **f** Dual-luciferase assays showed diminished luciferase activity was observed when co-transfection of psiCHECK-ULK1-WT and miR-20a-5p occurred in HEK 293 T and HPAF-II cells; **g** Luciferase reporter assay implied that decreased luciferase activity occurred in HEK 293 T and HPAF-II cells co-transfected with psiCHECK-PVT1-WT and miR-20a-5p compared with luciferase reporter with mutant type of PVT1 and miR-20a-5p; **h**, **i** qRT-PCR analysis of miR-20a-5p with augment (**h**) of PVT1 expression in Capan-2 and MIA PaCa-2 cells or attenuation (**i**) of PVT1 expression in SW1990 and HPAF-II cells; **j** Overexpression of miR-20a-5p made no contribution to the level of PVT1 expression. Data are presented as the mean ± S.D. (*n* = 3). ^*^P < 0.05, ^**^P < 0.01 by Student’s t-test

To understand whether the effect of miR-20a-5p on ULK1 was specific, we performed bioinformatics analysis and luciferase activity to detect whether miR-20a-5p was able to influence ULK1 expression. As shown in Fig. 7e-f, the luciferase reporter assay revealed that the wild-type 3’UTR of ULK1 showed low expression in the presence of miR-20a-5p, whereas the mutated 3’UTR did not show a significant response to miR-20a-5p. In addition, we tested whether PVT1 affects the activity of miR-20a-5p. MTS and colony formation assay indicated that cell proliferation capacity attenuated by overexpression of miR-20a-5p in Capan-2 cells was restored by up-regulation of PVT1. Also, cell proliferation potential enhanced by suppression of miR-20a-5p in HPAF-II cells was inhibited by down-regulation of PVT1 (Additional file 1: Figure S4a-b). Also, apoptosis promoted by up-regulation of miR-20a-5p was suppressed by increased expression of PVT1 (Additional file 1: Figure S4c). Bioinformatics analysis and luciferase activity assay showed that ectopic PVT1 expression counteracted the inhibitory effect of miR-20a-5p, whereas augmentation of miR-20a-5p had no effect on mutant PVT1, indicating that PVT1 can directly bind to miR-20a-5p (Fig. 7g). Besides, we did not observe obvious changes in miR-20a-5p levels following PVT1 overexpression (Fig. 7h) or knockdown (Fig. 7i). In addition, PVT1 expression was not altered after transfection with miR-20a-5p mimics (Fig. 7j). Taken together, these data suggest that PVT1 regulates ULK1 expression by sponging miR-20a-5p.

The article "LncRNA PVT1 triggers Cyto-protective autophagy and promotes pancreatic ductal adenocarcinoma development via the miR-20a-5p/ULK1 Axis" was retracted in 2022. Reasons: manipulated images; duplicated images; lack of ethics approval or compliance; a breach of policy by an author.

### PVT1 expression in PDA and its relationship with patient prognosis

To explore the relevance of PVT1 in PDA development, we first sought to determine the levels of PVT1 expression from the PDA patient cohorts in the Gene Expression Omnibus (GEO) database. An analysis of pancreatic cancer patient gene profiling results (GSE15471 and GSE16515) showed that PVT1 was more highly expressed in PDA tissues than in non-tumor tissues (Fig. 8a-b). To validate this phenomenon, we investigated PVT1 expression in 68 PDA tissues and their corresponding adjacent non-tumor tissues. As shown in Fig. 8c, PVT1 levels were elevated in 53 out of 68 PDA tissues compared with the corresponding non-tumor tissues. Moreover, the expression of PVT1 in high-grade (III + IV) PDA tissues was higher than that in low-grade (I + II) PDA tissues (Fig. 8d). Next, we examined the correlation between PVT1 expression and PDA patient prognosis. Kaplan-Meier survival analysis showed that the overall survival time for patients with high PVT1 expression was significantly shorter than that of patients with low PVT1 expression (Fig. 8e). To confirm the independent prognostic significance of PVT1, a multivariate analysis was performed to establish the relationship between PVT1 expression and clinical and pathological characteristics (Table 1). The results were consistent with previous findings in another cohort of patients [17] and suggested that PVT1 participated in PDA progression.

**Fig. 8:** PVT1 is up-regulated in PDA, correlates with PDA progression and predicts prognosis. **a**, **b** Data mining of PVT1 in PDA patients gene profiling GSE16515 (**a**) and GSE15471 (**b**). PVT1 is overexpressed in PDA tissues compared with the corresponding adjacent non-tumor pancreatic specimens. Data are presented as the mean ± S.D.. ^**^P < 0.001 by Student’s t-test; **c** PVT1 expression in 68 PDA patients. Fold change > 2 is used as the cut-off value in the expression. The high value of PVT1 was defined as fold change > 2 (*n* = 53), the rest was defined as low expression (*n* = 15); **d** PVT1 expression is up-regulated in patients with stage III + IV (*n* = 24) compared with patients with stage I + II (*n* = 44). Data are presented as the mean ± S.D.. ^*^P < 0.05 by Student’s t-test; **e** High expression of PVT1 predicts poor prognosis in 68 PDA patients. ^*^P < 0.05 by the log-rank test

**Table 1:** Clinicopathological characteristics of 68 pancreatic ductal adenocarcinoma patients

Clinicopathological parameters	Patients number	PVT1 expression		*P*-value^a^
		Low	High	
	68	15	53	
Gender				0.2467
Male	37	11	26	
Female	31	4	27	
Age (yr)				0.0956
<65	46	12	34	
≥65	22	3	19	
Tumor site				0.5981
Head	49	10	39	
Body+Tail	19	5	14	
Tumor size (cm)				0.8218
≤3	30	7	23	
>3	38	8	30	
Tumor classification				0.0425^*^
T1-T2	8	4	4	
T3-T4	60	11	49	
Lymph node metastasis				0.0209^*^
Absent	32	11	21	
Present	36	4	32	
Distant metastasis				0.1092
Absent	60	15	45	
Present	8	0	8	
Clinical stage (AJCC)				0.0086^*^
I-II	44	14	30	
III-IV	24	1	23	

^a^Chi-square test. ^*^P<0.05

## Discussion

In the present study, we have demonstrated that PVT1 is overexpressed and triggers protective autophagy in PDA cells by up-regulating ULK1 protein, which leads to the growth and progression of PDA in vitro and in vivo. Specifically, we found that PVT1 functions as a ceRNA by competing with endogenous miR-20a-5p, then elevates ULK1 protein expression (Fig. 9). These findings reveal a potential role for PVT1 in autophagy regulation and PDA cell growth.

The article "LncRNA PVT1 triggers Cyto-protective autophagy and promotes pancreatic ductal adenocarcinoma development via the miR-20a-5p/ULK1 Axis" was retracted in 2022. Reasons: manipulated images; duplicated images; lack of ethics approval or compliance; a breach of policy by an author.

**Fig. 9:** Schematic diagram shows the results of the study. PVT1 is up-regulated in PDA. Moreover, it triggers cyto-protective autophagy and promotes PDA cells growth and progression. It acts as a ceRNA to compete with miR-20a-5p, which leads to enhanced expression of ULK1, a key molecule involved in triggering autophagy initiation

Aberrant expression of some lncRNAs, such as MALAT1 [17], HOTTIP [32], H19 [33] and Mir31HG [34], has recently been reported to function in the tumorigenesis and progression of PDA. In the present study, qPCR analysis showed that PVT1 levels were significantly higher in PDA tissues than in the corresponding adjacent non-tumor tissues, in agreement with microarray gene expression profiling (GSE15471 and GSE16515) results. Similarly, compared with the immortalized pancreatic ductal epithelial cell line H6C7, PVT1 expression was strikingly higher in a panel of PDA cell lines, except for the Capan-2 and MIA PaCa-2 cell lines. In addition, higher levels of PVT1 closely correlated with advanced clinical stages and shorter survival in PDA patients, indicating that PVT1 acts as an oncogenic lncRNA in PDA [35].

Autophagy is a highly conserved self-degradative process that plays a key role in cellular stress responses and survival. Many cancers, including PDA, become dependent on autophagy as a source of nutrients during tumor growth [36, 37], previous reports have shown that PVT1 can participate in multiple biological processes crucial for PDA development, including proliferation [16], metastasis [17], and chemoresistance [19]. Despite the biological importance of PVT1, whether PVT1 is involved in the regulation of the autophagic program in PDA remains unclear. Besides, ULK1 is known to be a key molecule involved in triggering autophagy initiation and is regulated by amino acid and energy status via mTORC1 and AMPK [38, 39]. ULK1 expression is up-regulated in multiple tumor types and is associated with tumor progression and resistance to cancer chemotherapy [40–42]. First, we investigated the correlation between the expression level of ULK1 protein and PVT1. It is indicated that ULK1 protein levels parallel PVT1 expression in a subset of human PDA tissues. Interestingly, by examining our PDA tissues and two independent PDA cohorts from Oncomine, we found that ULK1 was up-regulated and correlated with PDA prognosis. In addition, applying gain-of-function and loss-of-function approaches, we demonstrated that PVT1 induces autophagy by up-regulating ULK1 protein both in vitro and in vivo. Thus, our study established that increases in ULK1 levels are due, in part, to induction of the oncogene PVT1, providing a possible mechanism for the up-regulation of ULK1 in PDA.

The article "LncRNA PVT1 triggers Cyto-protective autophagy and promotes pancreatic ductal adenocarcinoma development via the miR-20a-5p/ULK1 Axis" was retracted in 2022. Reasons: manipulated images; duplicated images; lack of ethics approval or compliance; a breach of policy by an author.

Previous studies have revealed that PVT1 interacts with c-Myc [12] or the proliferation-associated nucleolar protein NOP2 and stabilizes those proteins from degradation [16]. Recently, some lncRNAs have been reported to act as ‘sponges’ to bind specific miRNAs and regulate their function [23–25]. For example, the lncRNA HOTAIR functions as a ceRNA to increase the expression of HER2 via miR-331-3p and to drive gastric cancer growth and invasion [43]. The lncRNA HULC interacts with miR-372, thereby modulating PRKACB expression and activity in liver cancer [44]. In our present study, bioinformatics analysis revealed a healthy minimum free energy of hybridization between PVT1 and miR-20a-5p of − 26.2 kcal mol^− 1^. These results suggest that PVT1 is accessible to miR-20a-5p and that the interaction between PVT1 and miR-20a-5p is effective. Here, we provide evidence that PVT1 may also function as a sponge for miR-20a-5p, as miR-20a-5p levels were not affected following PVT1 knockdown or overexpression. We found that, similar to miR-20a-5p mimics, PVT1 down-regulation was able to suppress the miR-20a-5p target gene ULK1, whereas PVT1 up-regulation inhibited miR-20a-5p function, leading to derepression of ULK1. Therefore, the effect of PVT1 on PDA cell autophagy can be explained, at least in part, by its function as a molecular sponge for miR-20a-5p, providing a potential mechanism by which PVT1 acts as a tumor oncogene.

## Conclusion

In conclusion, the present study revealed that PVT1 was up-regulated in PDA tissues and cell lines. Higher levels of PVT1 were associated with tumor progression and were inversely correlated with prognosis. Knocking down PVT1 significantly suppressed cell autophagy and growth both in vitro and in vivo. Mechanistically, we provide the first evidence that PVT1 functions as a molecular sponge for miR-20a-5p to up-regulate ULK1. Our data provide a better understanding of the ceRNA network involving PTV1 in PDA progression. In addition, the “PVT1/miR-20a-5p/ULK1/autophagy” pathway is a novel target for developing therapeutic strategies to treat PDA.

## Additional files

Additional file 1: **Figure S1.** Expression pattern of ULK1 in a cohort of PDA patients in TCGA and cell lines. **Figure S2.** PVT1 regulates ULK1 expression in a posttranscriptional manner. **Figure S3.** Cellular location of PVT1 and miR-20a-5p in PDA cells. **Figure S4.** miR-20a-5p suppressed PVT1 function. **Table S1.** Clinicopathological information of 68 PDA patients in detail. **Table S2.** The PCR primer sequence to detect the target genes. **Table S3.** The sequence of the shRNAs to diminish the expression of PVT1. **Table S4.** Predicted microRNAs binding to ULK1 3’UTR by bioinformatics analysis. **Table S5.** Predicted microRNAs binding to PVT1 3’UTR by bioinformatics analysis. (ZIP 6594 kb)

The article "LncRNA PVT1 triggers Cyto-protective autophagy and promotes pancreatic ductal adenocarcinoma development via the miR-20a-5p/ULK1 Axis" was retracted in 2022. Reasons: manipulated images; duplicated images; lack of ethics approval or compliance; a breach of policy by an author.

## Abbreviations

ceRNAs: Competing endogenous RNAs
GEO: Gene expression omnibus
PDA: Pancreatic ductal adenocarcinoma
PVT1: Plasmacytoma variant translocation 1
RIP: RNA-binding protein immunoprecipitation
TCGA: The cancer genome atlas
ULK1: Unc-51 like kinase 1
